# Biomechanical Characteristics on the Lower Extremity of Three Typical Yoga Manoeuvres

**DOI:** 10.1155/2021/7464719

**Published:** 2021-08-12

**Authors:** Elizabeth Whissell, Lin Wang, Pan Li, Jing Xian Li, Zhen Wei

**Affiliations:** ^1^School of Human Kinetics, University of Ottawa, Ottawa, ON, Canada; ^2^School of Kinesiology, Shanghai University of Sport, Shanghai, China

## Abstract

This study was aimed at exploring the biomechanical characteristics of the lower extremity amongst three typical yoga manoeuvres. A total of thirteen experienced female yoga practitioners were recruited in the current study; they were all certified with the Yoga Alliance. A three-dimensional motion capture system with 10 cameras combined with four synchronised force plates was used to collect kinematics of the lower extremity and ground reactive force whilst the participants performed the crescent lunge pose, warrior II pose, and triangle pose. One-way repeated ANOVA was used in exploring the differences amongst the three yoga movements, and the significance was set to alpha < 0.05. The triangle pose performed the largest range of motion (ROM) of the hip (90.5° ± 22.9°), knee (68.8° ± 23.1°), and ankle (46.4° ± 11.3°) in the sagittal plane and the hip (54.8° ± 6.5°), knee (42.4° ± 12.8°), and ankle (4.8° ± 1.7°) in the frontal plane amongst the three manoeuvres (*P* < 0.05). No significant difference was found for the hip and ankle joint moment amongst the three manoeuvres (*P* > 0.05). Knee joint travelled into 9.5° of extension and slight adduction of 1.94° whilst expressing the largest knee joint adduction moments (0.30 ± 0.22 Nm/kg) in the triangle pose. The distribution of the angular impulse of the lower limb joints indicated that the hip joint contributed significantly the most in the sagittal and frontal planes of the three yoga manoeuvres (*P* < 0.05), ranging from 51.67% to 70.56%. Results indicated that triangle pose may be superior to the other two manoeuvres, which improved hip joint ROM, strength, and dynamic stability. However, knee injuries such as osteoarthritis (OA) should be considered because of the large knee extensor angle and adductor moments.

## 1. Introduction

Yoga is a mind-body exercise developed in India, which has gained popularity worldwide [1, 2]. This exercise can be characterised by slow movements, with large body movement range when participants are standing, seated, and lying supine or prone [3]. Practising yoga has been verified to increase muscle strength, joint flexibility [4], and joint range of motion (ROM) [5]; improve balance, coordination [6], and perceived stress and depression [2]; and reduce pain amongst patients with osteoarthritis (OA) [7].

Despite the potential benefits of yoga manoeuvres, yoga-related injuries should also be considered. Fishman et al. [8] have proposed that long-term incorrect yoga posture may result in lower back pain and lower limb muscle and ligament strain. Kuntz et al. [7] stated that yoga manoeuvres may affect the alignment of lower limb joints, which could contribute to knee injuries. Numerous studies in the current literature have explored the risk factors for yoga injuries, which could be related to poor yoga technique, incorrect joint alignment, previous injury history, excess effort, and insufficient instructions from the yoga instructor [8, 9]. Following to Mears et al. [5], by utilising a motion capture system and force plates to explore ankle ROM and moments in different yoga manoeuvres, studies on quantifying the kinematics and kinetics of yoga manoeuvres and exploring the possible mechanism of body yoga injuries are still lacking.

Raub and James [10] have described 57 basic yoga manoeuvres on the basis of traditional Iyengar yoga, of which several variations can be derived [11]. Different yoga manoeuvres could have different effects on the physical exercise and mechanism of injury [12]. As suggested by a previous study, Sauna yoga superiorly improves flexibility, strength, and balance [4]; alignment-based yoga exercise may be more efficacious for knee OA [7]. Even so, based on current reports, no study has been conducted to investigate the biomechanical difference of these typical yoga manoeuvres.

Therefore, the present study is aimed at exploring the biomechanical characteristics of the lower extremity amongst three representative yoga manoeuvres, namely, the crescent lunge pose (Halasana), warrior II pose (Virabhadrasana II), and triangle pose (Trikonasana). These three typical yoga manoeuvres are commonly found in various styles of yoga and are taught as introductory manoeuvres in many Hatha yoga classes for beginners and as an intermediary step to more advanced yoga manoeuvres [13, 14].

We hypothesise that the biomechanical characteristic of these yoga manoeuvres is different. The triangle pose may have a relatively higher maximum joint angle and moment, which are superior to the other two yoga manoeuvres, to improve lower limb joint angle and decrease lower extremity injury risk. The findings of the current study can contribute in determining the potential mechanisms of injury in yoga exercise and help participants improve their skills to prevent injuries.

## 2. Method

### 2.1. Participants

Thirteen experienced female yoga practitioners were recruited in the current study (aged 33.1 ± 5.40 years, body height 161.3 ± 5.6 cm, body mass 63.3 ± 10.4 kg, and practice experience 5.5 ± 1.05 years). These practitioners were all certified with a Yoga Alliance-accredited 200-hour Hatha yoga teacher-training course with a minimum of 5 years of teaching experience [15]. Participants would be excluded if they had musculoskeletal and/or other medical conditions in the previous 6 months before the study. The experiment was approved by the University Ethical Committee, and all participants signed an informed consent before the experiments.

### 2.2. Data Acquisition

All participants were asked to change into a skin-tight suit, and then, body height and body mass were measured. Forty-five reflective markers (14 mm diameter) were placed on anatomical landmarks of the participant in accordance to the Plug-in-Gait set [16]. The participants were given 10 min to warm up as they choose [17] (i.e., practice Sun Salutations or other yoga postures) and familiarise themselves with the data collection environment and protocols to ensure that participants move at a comfortable level of mobility.

A three-dimensional motion capture system with 10 cameras (Vicon MX-13, Oxford Metrics, Oxford, UK) was used to obtain marker trajectory with a sampling rate of 100 Hz. We synchronised four force platforms (Kistler 9287 C, Winterthur, Switzerland) embedded in the middle of the testing area in accordance to previous studies; the frequency of force plates was set at 1000 Hz [5, 18].

During data collection, practitioners were instructed to stand on the force plates, and a static calibration trial was recorded. In calibrating the system, the researcher would conduct a dynamic calibration using a T-shaped wand (240 mm) with three reflective markers. In practising a typical yoga manoeuvre and standardising the study, participants performed barefoot, and they were randomised in a counterbalanced order for three yoga manoeuvres. All the practices began from the downward dog and returned to the downward dog at their natural speed, and each practice was separated with a break consisting of five deep breaths in the downward dog (Figure 1).

### 2.3. Data Reduction and Statistical Analysis

The parameters for the right and left legs were collected, but only the data of the dominant leg were modelled to compute and analyse the required variables using Vicon Nexus (version 1.8, Oxford Metrics, Oxford, UK). The dominant leg was determined by kicking a ball [19]. Start and end of data collection were obtained as a motion cycle by inspecting the force vector emitted from the force plate and position of the virtual marker. Each motion cycle trial was time normalised on a time basis of 100% to mitigate the effect of the varying speed of each individual using a custom algorithm (MATLAB, MathWorks, Natick, USA) [20]. The angles in the sagittal and frontal planes were obtained by calculations derived from the Plug-in-Gait model, which predicted the joint centres of the hip, knee, and ankle in Vicon Nexus (v1.8) to find the maximum and minimum angles during each trial, and then, the ROM range was calculated. Raw kinetic data of the GRF from the force plates was filtered with a 6 Hz 2nd-order Butterworth low-pass filter. The kinematic data were modeled to compute the required variables with Vicon Nexus; the inverse dynamic model was utilised to calculate the kinetic parameters. The angular impulse was obtained by calculating the integral of the joint moment of each joint in the sagittal and frontal planes. It is expressed as the sum of the total angular impulse (Nm/kg) of one movement cycle. The profiles of the five successful normalised trials were averaged to obtain an ensemble average for each participant.

### 2.4. Statistical Analysis

All data were presented as mean and standard deviation. Shapiro–Wilk's test was used to test the normal distribution. One-way repeated ANOVA was used in exploring the differences amongst the three yoga movements. Bonferroni post hoc tests were conducted to compare specific differences. All variables were analysed using SPSS 22 software (SPSS Inc., Chicago, IL, USA). Statistical significance was set at alpha < 0.05.

## 3. Results

### 3.1. Lower Limb Joint Angle

The three yoga movements began in the same initial yoga posture, and all three joints in the frontal and sagittal planes began at the same joint angle (Table 1).

The ROM of the yoga movements was 90.5° for the hip, 83.3° for the knee, and 48.7° for the ankle in the sagittal plane and 54.8° for the hip, 44.9° for the knee, and 4.8° for the ankle in the frontal plane. When analysing the individual yoga movement, we observed that the triangle pose performed a significant and the largest ROM of the hip (90.5°), knee (68.8°), and ankle (46.4°) in the sagittal plane (*P* < 0.05) and hip (54.8°), knee (42.4°), and ankle (4.8°) in the frontal plane (*P* < 0.05) amongst the three yoga manoeuvres. Therefore, moving into the triangle pose required the most ROM for all three joints in both planes.

### 3.2. Lower Limb Joint Moment

#### 3.2.1. Sagittal Plane

No significant difference was found for the hip flexor moment throughout the entire movement cycle (*P* > 0.05): lunge (1.90 Nm/kg), warrior II (1.45 Nm/kg), and triangle (1.38 Nm/kg). Although the extensor moments were present in the knee joint, knee extension angles could only be achieved when practising the triangle pose, with 9.5° of extension. Furthermore, no plantar flexor moment was generated in any of the yoga movements (*P* > 0.05, Table 2).

#### 3.2.2. Frontal Plane

The hip joint adduction moments indicated that no significant difference was observed in the triangle (0.85 Nm/kg), lunge (0.69 Nm/kg), and warrior II (0.62 Nm/kg) (*P* > 0.05) poses. The knee joint in the triangle pose travelled into slight adduction of 1.94°, expressing the largest knee joint adduction moments (0.30 Nm/kg) compared with the lunge (0.06 Nm/kg) and warrior II (0.07 Nm/kg) poses. Notably, the triangle pose was the only posture that could generate remarkable knee adduction moment after the initiation of the movement at approximately 40% of the movement cycle. For ankle adductor moments and eversion moment, the peak value was similar amongst the three manoeuvres (*P* > 0.05), 0.06 Nm/kg for the warrior II pose and 0.07 Nm/kg for the lunge and triangle poses (Table 2).

### 3.3. Lower Limb Angular Impulses

Upon visual inspection distribution of the lower limb angular impulse, we found that the hip joint contributed significantly the most amongst the three studied yoga manoeuvres in the sagittal and frontal planes (*P* < 0.05), ranging from 51.67% to 70.56% of the total angular impulse. No significant difference was found for the ankle joint total angular impulse in the sagittal and frontal planes (*P* > 0.05). However, the knee shared the load differently in each individual posture (Table 3).

## 4. Discussion

This study is the first to quantitatively investigate three fundamental yoga manoeuvres by characterising the kinetics and kinematics associated with the hip, knee, and ankle joints amongst yoga practitioners. The findings demonstrated that the lunge and warrior II poses followed similar joint angle, joint moment, and angular impulse patterns, whereas the triangle pose obtained the largest ROM in all joints in the sagittal and frontal planes.

### 4.1. Lower Limb Joint Angle

When examining the yoga movement with regard to the joint angle pattern, limited ROM was observed in the knee and ankle joint angles between the lunge and warrior II poses. Notably, the knee joint reached a maximal flexion angle of 73.8° and 67.7° in the lunge and warrior II poses, respectively. These manoeuvres were typically described in yoga training manuals as having a 90° bend; therefore, the present study found that 16.2% to 22.3% was less than what was classically instructed in a yoga class. This result partially supported our hypothesis, which indicated that even experts did not perform the movement as it was ideally described and instructed.

Triangle pose practice was found to be distinct from the other selected poses as it expressed the largest ROM for all three joints in the sagittal and frontal planes. Practising the triangle pose caused the knee to extend over its baseline by 9.5° on average, and the increased extension has been shown to be significantly correlated to anterior cruciate ligament impingement in uninjured knees [21]. On the contrary, the hyperextension of the knee also contributed to the excessive strain on the oblique popliteal ligament and posterior cruciate ligament [22]. Therefore, even for yoga experts, it is important to avoid hyperextension and associated knee injuries during bending the knees in the triangle pose [9, 23].

Knee adduction angle could cause reduction in the patella cartilage volume in valgus knees amongst patients with OA [24]. We found that the knee joint in the triangle pose practice travelled into slight adduction of 1.9°, which was the only manoeuvre that showed knee adduction. Therefore, those who suffered from medial compartment knee OA should be cautioned during pursuing triangle yoga poses [25]. No increase in joint angles or moments was apparent for the ankle joint, indicating that the studied yoga postures did not improve the dynamic stability amongst the healthy participants who utilised ankle strategies for balance [26].

### 4.2. Lower Limb Joint Moment

Practising the triangle pose may also bring a concern to vulnerable populations, such as those who suffer from knee OA. Lower knee abductor moments could reduce knee pain, and the progression of knee OA increased 6.46 times with 1% increase in adduction moment [25]. Individuals with knee OA have significantly reduced isokinetic hip abductor strength. Those who suffered from knee OA increased hip abductor moment to protect against degeneration of the joint capsule [27]. However, no yoga manoeuvres, which were examined in the present study, showed hip abductor moments [28]. Therefore, examining manoeuvres with hip abductor moments or exploring various instructional words to encourage hip abductor strength in the triangle pose, reduce knee adduction moment, and protect those with knee OA is recommended in future studies.

Reduced lower limb abductor and adductor joint moments were also found to be prevalent in elderly people [29], and this reduced strength was associated with higher risks of falls [30]. The great hip adduction moments present in the yoga movements may suggest that the practice of yoga can be considered for future studies regarding training mechanisms that reduce falls, thereby improving dynamic stability [31].

On average, yoga expressed greater total hip ROM and hip flexor moments compared with activities of daily life (ADL) [3, 32], suggesting that yoga should be studied further as a potential training modality to improve daily gait [28, 33, 34]. In addition, the knee abduction angle and abductor moments were greater in yoga than in ADL [30]. Thus, this point should be kept in mind when considering yoga as a therapeutic or rehabilitation approach for knee joint disorders [35, 36].

Yoga solicits the hip joint moment in the frontal plane, which is associated with knee health and dynamic stability [37]. Future studies should focus on soliciting more abduction moments to promote overall knee health.

### 4.3. Lower Limb Angular Impulses

The hip contributed 51.67%–70.56% of the angular impulse in the lower limb in all three yoga movements compared with the knee and ankle, suggesting that yoga may have a strong training effect on the hip and may improve hip strength and ROM. Higher hip loading in yoga could be beneficial to those who rely on hip strategies for dynamic stability in gait [38, 39]. It is characterised by larger perturbation to the body movement, particularly by the sway in the hips. The finding is particularly interesting for elderly people who utilise the hip strategy during gait rather than ankle strategies [28]. Therefore, practising yoga should be recommended to the elderly to maintain postural stability [26], to those with the high possibility of fall [40], and to those with diabetes and peripheral neuropathy who suffer from impaired sensation in the ankles and feet [36, 41].

The ankle contribution in the sagittal plane represented approximately 26.27% of the contribution of the angular impulse. Ankle dorsiflexion and plantarflexion strength is negatively correlated with a history of falls in the elderly [26, 32, 39]. This finding further suggests that the elderly should consider practising yoga to improve postural stability for its potential application in hip and ankle strengthening amongst the elderly; however, it may not be sufficient in healthy individuals.

The present study has several limitations. Firstly, the motion pattern obtained from this study is only applicable for the lower extremity of healthy female yoga teachers. Secondly, when using eternal makers for the collection of motion capture, skin, clothing, and adipose tissue may cause artifact movement, thereby creating errors in the calculation of joint centres. Despite the above-mentioned possible limitations of this study, motion patterns of yoga movements could serve as a foundation for future applied research and clinical applications for people with disease.

## 5. Conclusion

The present study proposed that the lunge and warrior II poses shared similar motion patterns with regard to joint angles, joint moments, and angular impulse. The triangle pose may be superior to the other two manoeuvres, which improves hip joint ROM, strength, and dynamic stability. However, knee injuries such as OA should be paid attention to because of the large knee extensor and adductor moments. These findings will help practitioners when practising yoga by using scientifically based evidence.

## Figures and Tables

**Figure 1:** Three typical yoga manoeuvres.

**Table 1:** Mean and standard deviation for peak joint angles and range of motion (°) in the sagittal and frontal planes.

		Flex/ext			Abd/add		
		Max	Min	ROM	Max	Min	ROM
Yoga averages	Hip	121.3 ± 0.5	52.8 ± 27.2	90.5	−3.7 ± 3.2	−41.3 ± 28.7	54.8
	Knee	66.9 ± 7.3	17.1 ± 23.1	83.3	41.8 ± 1.3	13.3 ± 13.6	44.9
	Ankle	9.2 ± 1.2	−17.0 ± 18.4	48.7	5.8 ± 0.9	2.1 ± 0.3	4.8
Lunge	Hip	121.3 ± 10.4	83.3 ± 14.7	38.0 ± 13.1	−0.1 ± 5.1	−8.3 ± 5.3	8.2 ± 3.8
	Knee	73.8 ± 17.6	31.0 ± 18.0	42.7 ± 15.3	42.9 ± 15.0	17.6 ± 8.9	25.3 ± 12.7
	Ankle	9.1 ± 7.3	−6.6 ± 8.4	15.7 ± 7.2	4.8 ± 2.9	2.1 ± 2.5	2.8 ± 1.3
Warrior II	Hip	120.8 ± 12.6	43.8 ± 23.9	77.0 ± 24.3	−5.5 ± 6.0	−55.3 ± 6.4	49.7 ± 7.5
	Knee	67.7 ± 19.9	29.9 ± 15.7	37.8 ± 14.3	42.0 ± 8.9	24.2 ± 9.2	17.8 ± 9.9
	Ankle	10.4 ± 5.4	−6.3 ± 7.7	16.7 ± 6.5	6.0 ± 3.2	2.4 ± 2.6	3.6 ± 1.5
Triangle	Hip	121.8 ± 11.8	31.3 ± 22.8	90.5 ± 22.9^∗^	−5.5 ± 5.5	−60.3 ± 6.1	54.8 ± 6.5^∗^
	Knee	59.2 ± 23.5	−9.5 ± 6.1	68.8 ± 23.1^∗^	40.4 ± 12.2	−1.9 ± 5.4	42.4 ± 12.8^∗^
	Ankle	8.1 ± 9.2	−38.3 ± 7.5	46.4 ± 11.3^∗^	6.6 ± 3.0	1.8 ± 2.4	4.8 ± 1.7^∗^

Note: positive values indicate flexion and abduction and negative values indicate extension and adduction; significant differences (^∗^*P* < 0.05) are highlighted in bold.

**Table 2:** Mean and standard deviation of bodyweight-normalised peak joint moments (Nm/kg) in the sagittal and frontal planes.

		Flex/ext		Abd/add	
		Max	Min	Max	Min
Yoga averages	Hip	1.58 ± 0.28	0.08 ± 0.02	0.07 ± 0.03	−0.72 ± 0.12
	Knee	0.24 ± 0.14	−0.50 ± 0.38	0.37 ± 0.04	−0.14 ± 0.13
	Ankle	0.67 ± 0.11	0.03 ± 0.01	0.03 ± 0.00	−0.07 ± 0.00
Lunge	Hip	1.90 ± 0.34	0.07 ± 0.20	0.08 ± 0.09	−0.69 ± 0.46
	Knee	0.16 ± 0.20	−0.31 ± 0.15	0.33 ± 0.10	−0.06 ± 0.04
	Ankle	0.80 ± 0.11	0.04 ± 0.04	0.03 ± 0.32	−0.07 ± 0.02
Warrior II	Hip	1.45 ± 0.56	0.06 ± 0.19	0.09 ± 0.11	−0.62 ± 0.41
	Knee	0.40 ± 0.34	−0.25 ± 0.12	0.37 ± 0.17	−0.07 ± 0.06
	Ankle	0.61 ± 0.25	0.02 ± 0.03	0.03 ± 0.04	−0.06 ± 0.03
Triangle	Hip	1.38 ± 0.38	0.10 ± 0.10	0.03 ± 0.12	−0.85 ± 0.26
	Knee	0.16 ± 0.27	−0.94 ± 0.22	0.40 ± 0.21	−0.30 ± 0.22
	Ankle	0.61 ± 0.15	0.04 ± 0.04	0.02 ± 0.03	−0.07 ± 0.03

Note: positive values indicate flexion and abduction and negative values indicate extension and adduction.

**Table 3:** Mean and standard deviation of the total angular impulses (Nm) in the sagittal and frontal planes.

	Movement	Hip	Percent	Knee	Percent	Ankle	Percent
Yoga averages	Flex/ext	99.54	61.02%	20.74	12.71%	42.86	26.27%
	Abd/add	40.21	64.64%	20.18	32.44%	1.82	2.93%
Lunge	Flex/ext	132.35	68.35%	8.51	4.39%	52.78	27.26%
	Abd/add	34.41	61.36%	20.01	35.68%	1.66	2.96%
Warrior II	Flex/ext	83.64	61.56%	12.69	9.34%	39.53	29.10%
	Abd/add	34.83	60.35%	21.42	37.12%	1.46	2.53%
Triangle	Flex/ext	82.61	**51.67%** ^∗^	41.02	25.66%	36.26	22.68%
	Abd/add	51.4	**70.56%** ^∗^	19.12	26.25%	2.33	3.20%

Note: positive values indicate flexion and abduction and negative values indicate extension and adduction; significant differences (^∗^*P* < 0.05) are highlighted in bold.

## Data Availability

The datasets used and/or analysed during the current study are available from the corresponding authors upon reasonable request.
